# A Micro Neural Network for Healthcare Sensor Data Stream Classification in Sustainable and Smart Cities

**DOI:** 10.1155/2022/4270295

**Published:** 2022-06-24

**Authors:** Jin Wu, Le Sun, Dandan Peng, Siuly Siuly

**Affiliations:** ^1^Engineering Research Center of Digital Forensics, Ministry of Education, Nanjing University of Information Science and Technology, Nanjing, China; ^2^Department of Jiangsu Collaborative Innovation Center of Atmospheric Environment and Equipment Technology (CICAEET), Nanjing University of Information Science and Technology, Nanjing 210044, China; ^3^School of Computer Science and Network Engineering, Guangzhou University, Guangzhou, Guangdong, China; ^4^Centre for Applied Informatics, College of Engineering and Science, Victoria University, Melbourne, Australia

## Abstract

A smart city is an intelligent space, in which large amounts of data are collected and analyzed using low-cost sensors and automatic algorithms. The application of artificial intelligence and Internet of Things (IoT) technologies in electronic health (E-health) can efficiently promote the development of sustainable and smart cities. The IoT sensors and intelligent algorithms enable the remote monitoring and analyzing of the healthcare data of patients, which reduces the medical and travel expenses in cities. Existing deep learning-based methods for healthcare sensor data classification have made great achievements. However, these methods take much time and storage space for model training and inference. They are difficult to be deployed in small devices to classify the physiological signal of patients in real time. To solve the above problems, this paper proposes a micro time series classification model called the micro neural network (MicroNN). The proposed model is micro enough to be deployed on tiny edge devices. MicroNN can be applied to long-term physiological signal monitoring based on edge computing devices. We conduct comprehensive experiments to evaluate the classification accuracy and computation complexity of MicroNN. Experiment results show that MicroNN performs better than the state-of-the-art methods. The accuracies on the two datasets (MIT-BIH-AR and INCART) are 98.4% and 98.1%, respectively. Finally, we present an application to show how MicroNN can improve the development of sustainable and smart cities.

## 1. Introduction

International Telecommunication Union (ITU) and the United Nations Economic Commission for Europe (UNECE) jointly put forward the construction scheme of a sustainable smart city [1, 2]. The scheme aims to use information technology to improve the level of people's living standards and increase the efficiency of urban services [3]. Problems, such as uneven distribution of medical resources and low efficiency of disease treatment, have gradually become prominent in urban construction [4, 5]. Many research works [6, 7] explore advanced Internet of Things (IoT) and artificial intelligence technologies to solve these problems to promote the development of urban intelligence and sustainability.

The rapid development of deep learning technology and the Internet of Medical Things (IoMT) has brought new opportunities and challenges to medical development in the construction of smart cities [3]. In recent years, some algorithms [6, 8] based on deep learning have been proposed to classify healthcare sensor data streams to solve the problem of medical problems in the process of urban development. Deep convolution neural network (CNN) [9] and deep recurrent neural network (RNN) [10] are two popular methods for classifying healthcare sensor data streams. The former is mainly represented by the one-dimensional convolutional neural network, which can extract the features of one-dimensional time series data [11]. The latter mainly serializes the neurons to process the serialized data, so that the neurons among the hidden layers can be related to each other [10]. Most of the existing healthcare sensor data classification methods are improved based on the above two methods. However, these methods are difficult to deploy in edge devices because of their large time and space complexity [12].

To reduce the reasoning time and spatial complexity of the model, different lightweight neural network models are proposed in the literature [13, 14]. These methods can be divided into three scenarios: artificially designed lightweight neural network, neural network model compression algorithm, and automatic design of neural network structures [15]. In the first scenario, the model is made lightweight by reducing the number of parameters, for example, limiting the number of channels of features [16, 17], using decomposition convolution operation or 1*∗*1 convolution kernel [18], etc. However, the design process of this scenario needs a lot of time [19]. The second scenario mainly uses knowledge distillation [20] and network slimming [21] to compress the network model. Unfortunately, these methods often realize the lightweight of the model at the cost of sacrificing the performance of the model. The third scenario is to automatically design a neural network architecture to solve a specific task according to a certain search strategy [15, 22, 23]. When using the methods based on the above scenarios to classify healthcare sensor data streams, the accuracy of the models is not very high. It is mainly because these models do not consider how to distinguish classes with similar features [24, 25].

In contrast to the above methods, this paper proposes a novel model that ensures the classification accuracy of each class while ensuring the lightweight of the model, called MicroNN. Since RNN has the advantage of memory preservation for time series data, the architecture based on multilayered RNN [26] is used as the feature extractor of MicroNN. In addition, to improve the identification ability of MicroNN between classes with similar features [27], Kullback Leibler divergence (KL divergence) is introduced in this paper. Experiments show that the overall accuracy and the classification accuracy of each class using MicroNN exceed other work. Our main contributions are as follows:

- MicroNN model is composed of a microfeature extractor and some miniclassifiers.
- MicroNN uses a method based on KL divergence to eliminate shared knowledge among classes.
- We conduct comprehensive experiments based on time complexity and space complexity.

The rest of this paper is organized as follows: section 2 presents the related work, section 3 introduces the proposed model, section 4 shows the experiment, section 5 describes an application scenario of MicroNN, and section 6 summarizes this work.

## 2. Related Work

E-health has become a part of the development of sustainable and smart cities [2, 32]. With the mature development of deep learning and IoMT, healthcare sensor data stream classification based on edge computing has become possible [1, 33, 34]. It will effectively alleviate the uneven distribution of urban medical resources and further accelerate the intelligence development of cities.

According to the survey [6], different diseases are bothering mankind, which seriously threaten human life and quality of life. Nowadays, how to detect and avoid related diseases as soon as possible has become a major issue in urban development [1, 35]. Therefore, disease diagnosis based on healthcare sensor data stream classification has become a hot research topic. Many pieces of research use traditional machine learning methods to classify healthcare sensor data streams, which rely heavily on the characteristics of manual design. Behadada and Chikh [36] proposed a method based on the fuzzy decision tree to improve the detection of arrhythmias. Nasiri et al. [37] designed a model based on the support vector machine and genetic algorithms to diagnose cardiac arrhythmia with relatively high accuracy. Bensujin and Hubert [38] raised a method by combining the *K*-means clustering algorithm and bacterial foraging optimization algorithm to examine the heart situation of a person. Sharipov [39] used principal component analysis to improve the cardiac diagnosis via ECG. Jadhav et al. [40] proposed static backpropagation algorithms and the momentum learning rule for diagnosing heart diseases.

At present, because of the excellent performance of deep learning technology in the fields of image classification and text recognition, more research works are trying to apply the deep learning model in the field of disease diagnosis. Liu et al. [26] developed a model based on a multiple-feature-branch convolutional neural network for checking the patient's abnormal heartbeat. Chen et al. [28] proposed a new end-to-end scheme using a convolutional neural network (CNN) for automated ECG analysis. Saadatnejad et al. [30] proposed multiple long-short term memory (LSTM) models to monitor the status of heart activity. Faust et al. [31] proposed a bidirectional LSTM for beat detection. Jun et al. [29] used a CNN model with more layers by transforming the healthcare sensor data into a two-dimensional gray image.

Our work is different from the above work. In Table 1, we compare MicroNN with the discussed methods in terms of space complexity. It can be found that the space complexity of the models discussed is relatively larger than MicroNN. It makes some models not widely used in portable devices or edge devices. Therefore, this paper not only considers the accuracy of the model but also further considers the space complexity of the model (Table 2).

## 3. Our Proposed Model

### 3.1. System Overview

MicroNN mainly includes three parts: preprocessing model, microfeature extractor, and miniclassifiers.  Figure 1 shows the overall architecture of MicroNN. Table 2 is an explanation of the notations used in the paper. The workflow of MicroNN is as follows: a physiological information record *X*={*x*_1_, *x*_2_,…, *x*_*n*_}. The preprocessing model splits the record into slices with equal length *n*, and each slice refers to *S*_*i*_={*v*_1_, *v*_2_,…, *v*_*r*_}.

Then, the microfeature extractor is used to extract the features of *S*_*i*_, *F*_*i*_={*e*_1_, *e*_2_,…, *e*_*m*_}. Finally, the feature  *F*_*i*_ of *S*_*i*_ is input into each miniclassifier *f*_*i*_ to obtain the corresponding score. Hence, the label of heartbeat *S*_*i*_ is *y,* as shown in (1).

(1) $$\begin{array}{c} y=\arg\max_{i}\left(f_{1},f_{2},\ldots ,f_{n}\right). \end{array}$$

### 3.2. Preprocessing Model

Physiological signals are mainly measured by some mobile edge devices. However, as physiological signals have the characteristics of low amplitude and low frequency, it is easy to be disturbed by noise in the acquisition process [39]. These noises mainly come from internal or external interference [36]. Therefore, the wavelet transform [41] is used to denoise the original signal in this paper. Firstly, the original data is decomposed into nine scales. Then, the wavelet coefficients of nine scales will be processed by threshold operation [41]. Finally, we reconstruct the original data by inverse wavelet transform.  Figure 2 shows the changes in physiological signal records (such as ECG) before and after denoising. Secondly, each physiological signal record is segmented into slices based on the annotations provided by the standard file [42]. Each slice *S*_*i*_ was normalized, *S*_*i*,*j*_=*S*_*i*,*j*_/‖*S*_*i*_‖_2_, where *S*_*i*,*j*_ represents the *j* **th** point of *S*_*i*_ and ‖*S*_*i*_‖_2_ refers to the 2-norm of a heartbeat slice *S*_*i*_.

### 3.3. Microfeature Extractor and Miniclassifiers

In the past, many research works used the convolutional neural network (CNN) as a feature extraction model. However, as CNN needs more computing and storage resources [26], it is difficult to deploy it in edge devices. Consider that the recurrent neural network (RNN) has a memory function in the processing of medical time series data and that its volume is smaller than that of the convolutional neural network [28]. Inspired by ShaRNN [43], this paper mainly adopts the collection of multilevel RNNs as the feature extractor (see Figure 1).

Firstly, it should be noted that we set the RNN collection with two levels. We set the slice data after preprocessing as *S*_*i*_={*v*_1_, *v*_2_,…, *v*_*r*_}, and we will divide it into some slices whose size is *ω*. *S*_*i*_ will generate *n*/*ω* slices, and we use *A*_*k*_ to represent each slice. Then, we set up an RNN model for each slice:

(2) $$\begin{array}{c} \beta_{k}^{\left[1\right]}={\text{RNN}}^{\left[1\right]}\left(A_{k}\right),\;k\in \left[1,\frac{n}{\omega }\right]. \end{array}$$

Here, RNN^[1]^ represents the RNN model of the first level, and *β*_*k*_^[1]^ refers to the output of *k*^**th**^ slice by RNN^[1]^. Therefore, we can get the result [*β*_1_^[1]^, *β*_2_^[1]^,…, *β*_*n*/*ω*_^[1]^] after the training of RNNs collection of the first level.

In the next step, we feed the result into the RNN of the second level, and the output is

(3) $$\begin{array}{c} \beta^{\left[2\right]}={\text{RNN}}^{\left[2\right]}\left(\beta_{1}^{\left[1\right]},\beta_{2}^{\left[1\right]},\ldots ,\beta_{n/\omega }^{\left[1\right]}\right),\;y=ℱ\left(\beta^{\left[2\right]}\right), \end{array}$$

where RNN^[2]^ represents the RNN model of the second level, ℱ refers to the activation function, and *y* is the extracted feature. It should be noted that RNN^[1]^ or RNN^[2]^ can be any RNN model, such as RNN, LSTM, Bi-LSTM, GRU, and so on.

In the selection of a classifier for MicroNN, we adopt a per-class classification model. The model will establish a separate miniclassifier for each class of the task (see the part of classification in Figure 1). All miniclassifiers are connected with the feature extractor. In addition, to improve the performance of the classifier, we employ a loss function called one-class [24] in the training process:

(4) $$\begin{array}{c} \text{loss}=E_{X∼P_{X}^{{\text{class}}_{i}}}\left[-\log\left(\sigma \left(f_{i}\left(X\right)\right)\right)\right]+\eta \cdot E_{X∼P_{X}^{{\text{class}}_{i}}}{\left|\left|\frac{\partial f_{i}\left(X\right)}{\partial X}\right|\right|}_{2}^{c}+\pi \cdot {\left|\left|\theta_{i}-\mu_{1:i-1}^{*}\right|\right|}_{2}^{2}, \end{array}$$

where *X* ~ *P*_*X*_^class_*i*_^ refers to the data distribution of each class, *σ* is the activation function, and *η*, *c*, and *π* are all hyperparameters.

The first term in the loss function is negative log likelihood. Its purpose is to maximize the score of class_*i*_ during training. However, if there is no constraint to the negative log likelihood, it will lead to an unlimited increase in the score. Therefore, the second term, which is called *H*-reg, is applied in the loss function. It can reach a balance with the negative log likelihood. The structure of per-class classification is a multilayer perceptron with three layers, as shown in (5).

(5) $$\begin{array}{c} E_{X∼P_{X}^{{\text{class}}_{i}}}{\left|\left|\frac{\partial f_{i}\left(X\right)}{\partial X}\right|\right|}_{2}^{c}=E_{X∼P_{X}^{{\text{class}}_{i}}}{\left|\left|\frac{\partial W_{3}\cdot \left[\sigma \left(W_{2}\cdot \sigma \left(W_{1}\cdot X\right)\right)\right]}{\partial X}\right|\right|}_{2}^{c}. \end{array}$$

We can see that the derivation result of *H*-reg in the training process is related to the weight (*W*_1_,  *W*_2_ and *W*_3_). Therefore, *H*-reg can restrict the phenomenon of the unlimited growth of weight, which the negative log likelihood brings.

To make the parameters of classifiers between different classes in the same parameter space, the method uses the parameters from 1 to *i* − 1 miniclassifiers to initialize the parameters of the *i*^th^ miniclassifier. Considering the existence of similar features between different classes, deep learning models have difficulty distinguishing classes in the process of training. During the testing stage, a method based on KL-divergence [44] is used to reduce the shared knowledge between classes, as described in the third term of the loss function. Assuming that there are *T* miniclassifiers in MicroNN, the calculation of shared knowledge among *T* miniclassifiers is as shown in (6).

(6) $$\begin{array}{c} \rho_{1:T}^{*}=\arg\min\sum_{i=1}^{T}\varphi_{i}\text{ KL}\left(P_{i}\|P_{1:T}\right), \end{array}$$

where *φ*_*i*_ is the mixing ratio with ∑_*i*=1_^*T*^*φ*_*i*_=1, and *P*_*i*_ refers to the posterior parameter distribution of the *i*^th^ miniclassifier. The parameters of the *i*^th^ miniclassifier are updated by (7).

(7) $$\begin{array}{c} \vartheta_{i}^{*}=\vartheta_{i}-\tau \cdot \rho_{1:T}^{*}, \end{array}$$

where *τ* is a hyperparameter.

## 4. Performance Analysis

The experiments are conducted on a computer with a GPU of Intel (R) Core (TM) i9-11900K and 64.00 GB memory. Experiments are done on two different ECG datasets to evaluate the performance of MicroNN. In the experiment, we divide each dataset into training sets, validation sets, and test sets, and their proportions are 6 : 2 : 2, respectively. To better evaluate the performance of the model, we mainly use precision (Pre), recall (Rec), and *F*1-score (*F*1) in the paper. Their relationship is as follows:

(8) $$\begin{array}{c} F1=\frac{2\cdot \text{Pre}\cdot \text{Rec}}{\text{Pre}+\text{Rec}}. \end{array}$$

### 4.1. Datasets Description

The details of the two datasets used in the experiment are as follows:

1. MIT-BIH arrhythmia database (MIT-BIH-AR) includes the ECG record of 47 subjects studied by the BIH arrhythmia laboratory, and the sampling rate is 360 Hz. It contains 48 half-hour excerpts of two-channel ambulatory ECG recordings. In the experiment, we use the ECG record based on the MLII lead of MIT-BIH-AR. The full name of MIT-BIH is Massachusetts Institute of Technology, Beth Israel Hospital [42].
2. St Petersburg INCART 12-lead arrhythmia database (INCART) consists of 75 annotated records from 32 humans, and the sampling rate is 257 Hz. Each record lasts for a half-hour and has the data of 12 standard leads. In the experiment, we use the ECG record based on the II lead of INCART.

### 4.2. Performance of MicroNN

At first, we compared the performance of MicroNN with existing methods at MIT-BIH-AR and INCART (see Tables 3 and 4). Micro has achieved good performance in ACC and *F*1. As can be seen from Table 3, the low accuracy of other methods is mainly because of the low *F*1 of class *S*. It is because class *N* and class *S* have many similar characteristics. The model is prone to recognition errors. However, MicroNN ′s *F*1 in class *S* is much higher than other methods, which shows that MicroNN effectively reduces the shared knowledge among classes during training. Similarly, we can see from Table 4 that although the performance of MicroNN in classes *N* and *V* is not as good as partial work, MicroNN far exceeds other work in the classification of class *S*. It is mainly because that MicroNN can effectively solve the problem of the fuzzy boundary.

### 4.3. Measuring Time and Space Complexity of MicroNN

Table 2 compares the space complexity of MicroNN with other work, which shows that MicroNN is lightweight in terms of space complexity. In addition, we also measure the trend of training time and accuracy of MicroNN based on the change in the number of sample numbers in MIT-BIH-AR and INCART.

It can be seen from Figures 3 and 4 that the accuracy and training time of MicroNN increase with the increase of the number of instances of different datasets on the whole. In MIT-BIH-AR, when the number of instances reaches about 4000, the accuracy reaches 98.4% and tends to be stable. The training time is 23 seconds. For INCART, the number of instances reaches up to 4300 approximately, corresponding to the highest accuracy (98.1%), and the time of training is 27 seconds.

### 4.4. Threats to Validity

In the paper, threats to the validity of our proposed method are discussed from two perspectives: external validity and internal validity [14].

1. Threats to internal validity: To prevent the occurrence of overfitting, we divide each dataset into a training set, validation set, and test set. We observed the change in classification accuracy based on different validation sets to check whether the classification model has overfitting.
2. Threats to external validity: To verify the generalization of the model, we compared MicroNN on two different datasets. The experimental results show that the performance of MicroNN is better than other models.

## 5. An Engineering Application of MicroNN

Deep learning research on healthcare sensor data stream classification has attracted extensive attention [33, 54, 55]. However, we still face many challenges in the process of development. For example, the current urban medical resources are insufficient compared with the soaring urban population. The treatment efficiency cannot meet the needs of patients in time [4].

In this paper, we deploy MicroNN in edge devices to effectively improve the efficiency of medical treatment.  Figure 5 shows an application example of MicroNN based on edge computing. Different healthcare devices have the function of classifying healthcare sensor data streams. The healthcare devices will classify the collected physiological signals of patients. Then, the results will be used to assist doctors in judging the condition of patients. Finally, the doctor will inform the patient of the specific situation. Therefore, MicroNN plays a certain role in promoting the development of sustainable and smart cities.

## 6. Conclusion and Future Work

In this paper, we propose a lightweight neural network model called MicroNN for classifying healthcare sensor data streams. It is composed of a microfeature extractor based on multiple recurrent neural networks (RNNs) and multiple miniclassifiers based on a full connection layer with three layers. At the same time, the method based on KL divergence is used to remove the shared knowledge among different classes to improve the performance of the model. In the experiment, we compared the accuracy, time complexity, and space complexity of the model with other models based on two different ECG datasets. MicroNN shows better performance than other works. In a word, MicroNN is a lightweight and efficient model. We will further improve the accuracy of MicroNN while ensuring the lightweight of the model and extend experiments on other healthcare sensor datasets.

## Figures and Tables

**Figure 1:** The workflow of MicroNN.

**Figure 2:** The changes in a physiological signal record represented by ECG before and after denoising. (a) ECG record before denoising. (b) ECG record after denoising.

**Figure 3:** Accuracy with respect to the instance numbers in MIT-BIH-AR and INCART.

**Figure 4:** Time with respect to the instance numbers in MIT-BIH-AR and INCART.

**Figure 5:** An application of MicroNN on the Internet of Medical Things based on edge computing.

**Table 1:** The space complexity comparison between MicroNN and state-of-the-art methods.

Work	Methods	Model size (MB)
Liu et al. [26]	CNN	39.5
Chen et al. [28]	CNN	32.9
Jun et al. [29]	LSTM	16.2
Saadatnejad et al. [30]	LSTM	15.4
Faust et al. [31]	Bi-LSTM	27.6
Ours	MicroNN	13.7

**Table 2:** Meaning of the main notations.

Notation	Meaning
*X*={*x*_1_, *x*_2_,…, *x*_*n*_}	The raw physiological information record, *n* is the length of the record.
*S*_*i*_={*v*_1_, *v*_2_,…, *v*_*r*_}	*S*_*i*_ refers to the *i*^th^ slice after being segmented.
*S*_*i*,*j*_	*S*_*i*,*j*_ represents the *j*^th^ point of i^th^ slice.
*F*_*i*_={*e*_1_, *e*_2_,…, *e*_*m*_}	The features after feature extractor.
RNN^[1]^ , RNN^[2]^	RNN^[1]^ represents the collection of the RNN model at the first level, RNN^[2]^ represents the collection of the RNN model at the second level.
*X* ~ *P*_*X*_^class_*i*_^	It refers to the data distribution of each class.
*W*_1_, *W*_2_, and *W*_3_	They are the weights of a miniclassifier.
*f*_1_, *f*_2_,…, *f*_*n*_	They are the output of the miniclassifier.
*η* , *c* , and *π*	They are all hyperparameters in the paper.

**Table 3:** The performance comparison between MicroNN and state-of-the-art methods based on MIT-BIH-AR.

Work	Overall ACC(%)	*N* (%)			*S* (%)			*V* (%)		
		PRE	REC	*F*1	PRE	REC	*F*1	PRE	REC	*F*1
MicroNN	98.4	99.0	99.2	99.1	95.1	93.3	94.2	96.5	97.3	96.8
Llamedo and Martinez [45]	78.0	99.1	78.0	87.3	41.0	76.0	53.3	88.0	83.0	85.4
De Chazal et al. [46]	81.9	99.2	86.9	92.6	38.5	75.9	51.1	81.9	77.7	80.0
He et al. [47]	95.1	97.6	97.5	97.6	59.4	83.8	69.5	90.2	80.4	85.0
Zhai and Tin [48]	97.6	98.5	97.6	98.0	74.0	76.8	75.4	92.4	93.8	93.1
Lee et al. [49]	98.1	99.6	97.4	98.5	77.6	91.5	84.0	86.0	89.2	87.6
Li et al. [50]	98.1	98.0	99.8	98.9	94.7	68.7	79.6	91.1	95.5	93.2
Niu et al. [51]	97.5	97.4	98.9	98.1	76.6	76.5	76.5	94.1	85.7	89.7

**Table 4:** The performance comparison between MicroNN and state-of-the-art methods based on INCART.

Work	Overall ACC(%)	*N* (%)			*S* (%)			*V* (%)		
		PRE	REC	*F*1	PRE	REC	*F*1	PRE	REC	*F*1
MicroNN	98.1	99.0	99.0	99.0	88.3	91.1	85.6	95.5	95.0	95.2
Merdjanovska and Rashkovska [52]	94.3	97.7	93.8	95.7	69.3	75.0	72.0	95.7	86.1	90.6
Bidias àMougoufan et al. [53]	81.9	97.7	95.9	96.8	61.8	80.8	70.0	60.9	69.1	64.7
Sun et al. [42]	99.7	99.7	100	99.8	60.8	90.2	72.7	99.0	94.2	96.5

## Data Availability

The labeled datasets used to support the findings of this study are available from the corresponding author upon request.
